# *SLC39A8* gene encoding a metal ion transporter: discovery and bench to bedside

**DOI:** 10.1186/s40246-019-0233-3

**Published:** 2019-09-14

**Authors:** Daniel W. Nebert, Zijuan Liu

**Affiliations:** 1 Department of Environmental Health and Center for Environmental Genetics, University of Cincinnati Medical Center, Cincinnati, OH 45267-0056 USA; 2 Division of Human Genetics, Department of Pediatrics & Molecular Developmental Biology, Cincinnati Children’s Hospital, Cincinnati, OH 45229-2899 USA; 3 Department of Biological Sciences, Oakland University, Rochester, MI 48309 USA

**Keywords:** ZIP8 transporter, *SLC39A8* gene, Manganese uptake, Zinc uptake, Iron uptake, Selenium uptake, Genome-wide association studies, Cardiovascular disease, Schizophrenia, Type II congenital disorder of glycosylation, Leigh syndrome-like mitochondrial redox deficiency, Parkinson disease, Crohn disease, Pleiotropy

## Abstract

*SLC39A8* is an evolutionarily highly conserved gene that encodes the ZIP8 metal cation transporter in all vertebrates. *SLC39A8* is ubiquitously expressed, including pluripotent embryonic stem cells; *SLC39A8* expression occurs in every cell type examined. Uptake of ZIP8-mediated Mn^2+^, Zn^2+^, Fe^2+^, Se^4+^, and Co^2+^ represents endogenous functions—moving these cations into the cell. By way of mouse genetic differences, the phenotype of “subcutaneous cadmium-induced testicular necrosis” was assigned to the *Cdm* locus in the 1970s. This led to identification of the mouse *Slc39a8* gene, its most closely related *Slc39a14* gene, and creation of *Slc39a8*-overexpressing, *Slc39a8*(*neo*/*neo*) knockdown, and cell type-specific conditional knockout mouse lines; the *Slc39a8(−/−)* global knockout mouse is early-embryolethal. *Slc39a8*(*neo*/*neo*) hypomorphs die between gestational day 16.5 and postnatal day 1—exhibiting severe anemia, dysregulated hematopoiesis, hypoplastic spleen, dysorganogenesis, stunted growth, and hypomorphic limbs. Not surprisingly, genome-wide association studies subsequently revealed human *SLC39A8*-deficiency variants exhibiting striking pleiotropy—defects correlated with clinical disorders in virtually every organ, tissue, and cell-type: numerous developmental and congenital disorders, the immune system, cardiovascular system, kidney, lung, liver, coagulation system, central nervous system, musculoskeletal system, eye, and gastrointestinal tract. Traits with which *SLC39A8*-deficiency variants are currently associated include Mn^2+^-deficient hypoglycosylation; numerous birth defects; Leigh syndrome-like mitochondrial redox deficiency; decreased serum high-density lipoprotein-cholesterol levels; increased body mass index; greater risk of coronary artery disease, hypotension, cardiovascular death, allergy, ischemic stroke, schizophrenia, Parkinson disease, inflammatory bowel disease, Crohn disease, myopia, and adolescent idiopathic scoliosis; systemic lupus erythematosus with primary Sjögren syndrome; decreased height; and inadvertent participation in the inflammatory progression of osteoarthritis.

## Introduction

It could be said that “the *SLC39A8* story began in 1919,” when cadmium (Cd^2+^; Cd), administered subcutaneously to the rat, was shown to cause acute testicular necrosis without overt toxic effects in other organs. During the 1960s, inbred mouse strains were shown to differ in phenotype—most exhibiting “Cd-sensitivity,” but some showing “Cd-resistance.” In the 1970s, the mouse cadmium-responsiveness “*Cdm* locus” was defined.

Taking advantage of the latest advances in molecular biology techniques, it then became possible to identify unequivocally the mouse gene primarily responsible for the Cd-responsiveness trait. The gene was then realized to be evolutionarily highly conserved between mouse and other vertebrates including human. Not long after thoroughly characterizing functions of the gene product in mouse, genome-wide association studies (GWAS) began to appear, identifying clinical associations of minor allelic variants of the human gene encoding a deficient transporter—with an increasing array of disorders, physiological functions, and quantitative traits.

The present review details chronologically the century-long “bench-to-bedside” journey of this clinically important metal cation influx transporter. Roughly, this review is divided into two parts: first, early mouse studies that introduce the fundamental importance of this transporter involving many critical cellular functions; second, the numerous clinical disorders and quantitative traits with which the deficient transporter is correlated. Due to elucidation of the transporter in earlier mouse studies—many of the associated clinical disorders and phenotypes subsequently made more sense.

## Early Mouse *SLC39A8* Studies

### Original toxicity studies

Throughout the twentieth century, Cd was known to cause toxicity in laboratory animals and humans; however, no genetic or molecular mechanism of this trait was understood. In 1919, it was reported [1] that a single small dose of CdCl_2_—administered subcutaneously to rats—caused profound testicular damage within 24–48 h, while having no overt effect on other organs [2]. Furthermore, the Cd-induced-toxicity phenotype was found specifically to affect seminiferous tubular endothelial cells of testis, and the toxic response was shown to be similar across all vertebrates with testes—including rat, mouse, opossum, armadillo, pigeon, rooster, frog, and fish [3]. These data strongly suggested that “Cd-sensitivity” is the wild-type trait.

### Identification of the mouse *Slc39a8* gene

A subset of inbred strains of mice was discovered to be resistant to Cd-induced testicular necrosis [4]. Taylor and coworkers then demonstrated that Cd-sensitivity causing mouse testis damage is inherited as an autosomal dominant trait, and Cd-resistance is autosomal recessive [5]; the *Cdm* locus was mapped to a ∼24.6-cM segment on chromosome (Chr) 3 [6]. Two decades later, the Nebert lab [7] used polymorphic microsatellite markers and quantitative histological parameters to (a) corroborate the original 1973 data regarding Mendelian inheritance, and (b) refine the *Cdm* locus-containing region from more than 24 cM to 0.64 cM (which represented ~4.96 Mb). This was accomplished by phenotyping several inbred mouse lines—including C57BL/6 J (B6; Cd-resistant) and DBA/2 J (D2; Cd-sensitive)—plus the B6D2F_1_ heterozygote, and 26 BXD recombinant-inbred (RI) lines [7].

Next, single-nucleotide variant (SNV; also called “single-nucleotide polymorphism,” SNP) analysis of the 4.96-Mb region in two Cd-sensitive and two Cd-resistant mouse inbred strains, as well as in the BXD14/Ty RI line, revealed a 400-kb haplotype block associated with the Cd-toxicity phenotype [8]. Within this block was the *Slc39a8* gene—encoding a member of the solute-carrier (SLC) superfamily; at that time, the only homologous genes in the DNA database were those encoding a putative zinc-responsive (ZRT)-, iron-responsive transporter (IRT)-like Protein (ZIP) in plant and yeast genomes. Intriguingly, by means of in situ hybridization, *ZIP8* mRNA expression was strikingly elevated in the testicular vascular endothelial cells of Cd-sensitive, but not Cd-resistant, strains of mice [8].

If a function of the plant and yeast homologs is to transport Zn^2+^ or Fe^2+^, it was hypothesized that the mouse *Slc39a8* gene product would be a credible candidate for Cd^2+^ transport. In other words—if the function of ZIP8 is to move Cd into the cell, and it was well known that Cd must be intracellular in order to cause toxicity—then ZIP8 is a feasible candidate for explaining the Cd-induced testicular necrosis trait.

The *SLC* group now includes 66 gene families, comprising more than 400 protein-coding genes in the human and mouse genomes (https://www.genenames.org/). SLC proteins represent passive transporters, symporters, and antiporters—located in all cellular and organelle membranes of all vertebrates. Transport substrates include innumerable inorganic cations and anions, NH_4_^**+**^, amino acids and oligopeptides, glucose and other sugars, bile salts, carboxylate and other organic anions, acetyl coenzyme A, biogenic amines, neurotransmitters, vitamins, fatty acids and lipids, nucleosides, choline, thyroid hormone, and urea (reviewed in [9, 10]).

### Generation of a *Slc39a8*-overexpressing mouse line

A transgenic mouse line was created; this line carries a bacterial artificial chromosome (BAC) containing the *Slc39a8* gene from a 129/SvJ “Cd-sensitive” mouse, which had been inserted into the “Cd-resistant” B6 mouse genome [11]. This BAC-transgenic mouse (*BTZIP8*-*3*) genome was found to carry five *Slc39a8* gene copies—three from the BAC, plus the two wild-type diploid copies. ZIP8 expression was found to be highest in kidney, lung, and testis—but ubiquitously expressed to varying degrees throughout the animal [11]. In *BTZIP8*-*3* mice, when compared with wild-type B6 littermates, *ZIP8* mRNA and ZIP8 protein levels were shown to be expressed in these same tissues, but roughly 2.5-times higher in the *BTZIP8*-*3* line. Cd treatment failed to cause toxicity in nontransgenic littermates (which have the Cd-resistant B6 mouse genome), whereas Cd-induced testicular necrosis was seen in *BTZIP8*-*3* mice. Reversal of the trait—from Cd-resistance (in the host genome) to Cd-sensitivity in the BAC-carrying *BTZIP8*-*3* mouse—therefore confirmed unequivocally that the *Slc39a8* gene represents the *Cdm* locus [11].

### Characterization of the *Slc39a8*-encoding ZIP8 protein

Via stable retroviral infection, B6 ZIP8 cDNA was inserted into mouse fetal fibroblast cultures to create rvZIP8 cells; these stably transformed cultures revealed that ZIP8 expression is correlated with large increases in Cd^2+^ influx, intracellular accumulation, and Cd-induced cytotoxicity [12]. These cells were convenient for studying divalent cation uptake kinetics and Km values: Mn^2+^, more so than Zn^2+^, was determined to be the best physiological substrate for ZIP8 [12]. Subsequently, Fe^2+^ and Co^2+^ were also reported as ZIP8 substrates [13]. The ZIP8 protein is expressed in every mammalian tissue that has been examined (https://www.proteinatlas.org/ENSG00000138821-SLC39A8/tissue).

In ZIP8-expressing *Xenopus* oocyte cultures [14], electrogenicity studies showed an influx of two HCO_3_^**−**^ anions per one Zn^2+^ (or one Mn^2+^, or one Cd^2+^); these data imply that the complex moving across the cell membrane is a M^2+^/(HCO_3_^**−**^)_2_ electroneutral species. Subsequently, intracellular influx of selenite (HSeO_3_^−^)—an inorganic form of selenium having pharmaceutical importance—was demonstrated to depend on ZIP8, Zn^2+^, and HCO_3_^−^; thus, Zn^2+^/(HCO_3_^−^)(HSeO_3_^−^) was proposed as the most likely electroneutral complex [15].

### Membrane localization of ZIP8

Following Zn^2+^ treatment of cell cultures, the ZIP8 eight-transmembrane protein—under physiological Zn concentrations in the culture medium—was shown to be largely internalized; in contrast, under conditions of Zn^2+^ depletion in the medium, ZIP8 protein is trafficked predominantly to the cell-surface membrane [14]. In addition, ZIP8 transporter protein is known to be located in the plasma membrane that surrounds the intracellular organelles [12, 13], Golgi body [16, 17], lysosomal membrane [18], endoplasmic reticulum [19], and mitochondrial membrane [20].

### Identification and characterization of *SLC39A8*’s closest relative, *SLC39A14*

By alignment of amino acid sequences among the mouse *Slc39* gene subfamily of 14 members, it was found that *Slc39a14* was evolutionarily most closely related to *Slc39a8*; the *Slc39a14* gene was subsequently cloned and characterized [21]. *Slc39a14* expression is highest in liver > duodenum > kidney/brain > testis [21], whereas *Slc39a8* expression is highest in kidney > lung > testis [11]. By means of Z-stack confocal microscopy in transiently transfected Madin-Darby canine kidney (MDCK) polarized epithelial cells, the ZIP14 protein was demonstrated to be localized on the apical surface [21]—which is the same as that previously shown for ZIP8 [12]. Additionally, like ZIP8 [14], the ZIP14 protein was shown to be posttranslationally glycosylated [21].

The various similarities and many differences between the mouse *Slc39a8* and *Slc39a14* genes, human *SLC39A8* and *SLC39A14* genes, mouse ZIP8 and ZIP14 proteins, and human ZIP8 and ZIP14 proteins have been reviewed; please refer to the Table 1 of ref. [22].

### Evolutionary conservation of *SLC39A8*

Alignment of human and mouse *SLC39* members showed a very high degree of evolutionary conservation between each of the 14 orthologs [22]. This discovery strongly suggests that these 14 *SLC39* genes have existed for at least the last 80 million years and are likely to be critical to fundamental life processes. Because Cd-mediated testicular necrosis was noted in frog and fish [3]—it is highly likely that *SLC39A8* is present not only in all homeotherms, but all vertebrates. Moreover, *Slc39a8* is expressed in mouse gastrula [23], and visceral endoderm [24] at gestational day (GD)7.5; in fact, *SLC39A8* was proposed [25] as an indicator of cell differentiation (self-renewal-related signaling) in embryonic stem (ES) cells. These data strongly suggest that *SLC39A8*’s functions are critical from early embryogenesis, as well as later in adult life. Because *SLC39A14* is not expressed in ES cells, this is very strong evolutionary evidence supporting the likelihood that *SLC39A14* has arisen from a gene-duplication event from the earlier gene, *SLC39A8*.

### Original generation of *Slc39a8* knockout and knockdown mice

Given this information, it was hypothesized that a mouse *Slc39a8(−/−)* global knockout would likely be early-embryolethal. Subsequently, this was confirmed; no *Slc39a8(−/−)* global knockout embryo remnants were detected in utero at GD11.5 [26].

During attempts to create the global knockout, however, an interesting “knockdown” allele was serendipitously created. With *lox*P sites inserted into introns 3 and 6, the *lox*P-flanked segment was not removed by Cre recombinase, as intended; thus, the *Slc39a8(neo)* allele retained the (inversely oriented) *Frt*-flanked neomycin-resistance (*neo*) mini-cassette in intron 3 [26]. Intriguingly, *Slc39a8*(*neo*) was found to be a hypomorphic allele [26]: when compared to *Slc39a8(+/+)* wild-type, *Slc39a8*(*neo*/*neo*) homozygotes exhibit dramatically decreased *Slc39a8* mRNA and ZIP8 protein expression (~15% of that in wild-type yolk sac, and in every embryonic and fetal tissue examined). Yet, the *Slc39a8*(*neo*/*neo*) homozygote (having >99.8% B6 genetic background) remained viable—at least until GD16.5, with some pups surviving until postnatal day 1. Here, then, was an experimental model that provided a “window of time” for studying ZIP8 function in placenta, yolk sac, and fetal tissues.

### Phenotype of the *Slc39a8*(*neo*/*neo*) hypomorph

The *Slc39a8*(*neo*) allele is associated with diminished intracellular Mn^2+^, Zn^2+^, and Fe^2+^ in mouse fetal fibroblasts and liver-derived *Slc39a8*(*neo*/*neo*) cultures; levels of these endogenous cations are also decreased in several *Slc39a8*(*neo*/*neo*) newborn tissues [27]. Moreover, *Slc39a8*(*neo*/*neo*) homozygotes—from GD11.5 until death—are extremely pale and exhibit stunted growth and hypomorphic limbs. Additional abnormalities include a strikingly hypoplastic spleen and substantially reduced sizes of liver, kidney, lung, and brain (cerebrum, especially cerebellum). Histologically, *Slc39a8*(*neo*/*neo*) fetuses and neonates show decreased numbers of hematopoietic islands in yolk sac and liver; low hemoglobin levels, hematocrit, red cell count, serum iron, and total iron-binding capacity—everything consistent with the presence of severe anemia [27].

In an attempt to explain the *Slc39a8*(*neo*/*neo*) pleiotropy, bioinformatics analysis of the transcriptome was performed in GD13.5 yolk sac and placenta, as well as in GD16.5 liver, kidney, lung, heart, and cerebellum; *Slc39a8*(*neo*/*neo*) were compared with *Slc39a8(+/+)* wild-type mice [28]. Based on transcription factor profiles and searching for enriched transcription factor-binding sites, numerous genes encoding zinc-finger and other transcription factors associated with hematopoietic stem-cell functions were most prominent. It was concluded that in *Slc39a8*(*neo*/*neo*) mice, deficient ZIP8-mediated divalent cation transport—predominantly in GD13.5 yolk sac—affects zinc-finger transcription factors (such as GATA) and other transcription factors that interact with GATA proteins (such as the basic helix–loop–helix (bHLH) TAL1); among numerous other developmental functions, GATA proteins and TAL1 are well known to play critical roles in hematopoiesis. These RNA-seq data [28] thus strongly supported the in-utero pleiotropic phenotypes of dysregulated hematopoietic stem-cell fate, severe anemia, dysmorphogenesis, and underdeveloped organs of *Slc39a8*(*neo*/*neo*) mice [27].

Single-cell RNA-sequencing (scRNA-seq) studies have expanded our understanding of cellular diversification during gastrulation and early organogenesis; scRNA-seq profiles were generated from whole-mouse embryos collected at 6-h intervals between GD6.5 and GD8.5 [29]. In mice, this 48-h window is known to encompass key phases of gastrulation and early organogenesis—when pluripotent epiblasts are differentiating into ectodermal, mesodermal, and endodermal progenitors of all organs [30]. Pijuan-Sala et al. constructed a molecular map of cellular divergence from pluripotency toward all major embryonic lineages [29]. The pivotal role of TAL1 had previously been demonstrated in hematopoiesis [31]; in those experiments, *Tal1*(*−*/*−*) global knockout mouse embryos died with severe anemia around GD5.0. Therefore, by means of single-cell profiling, *Tal1*(*−*/*−*) chimeric embryos were generated, which showed defects in early mesoderm diversification [29]; these findings are consistent with the TAL1 deficiency-associated severe anemia and dysorganogenesis phenotypes seen in the *Slc39a8*(*neo*/*neo*) mouse [28], as detailed earlier.

Finding “an association,” however, does not imply any direct SLC39A8/TAL1 molecular interaction. There still might exist, say, two, or even 20, steps between ZIP8-mediated Zn (or other cation) intracellular uptake and TAL1 actions.

### Regulation of transporters in knockout and knockdown animals

Intriguingly, 29 differentially expressed *Slc* genes were found in the *Slc39a8*(*neo*/*neo*) transcriptomics analysis; some were prominent in two or three of the seven tissues examined, but most of them were differentially expressed in just one tissue [28]. Twenty-one of the 66 *Slc* gene families were represented, but none of the 14 genes in the *Slc39* family other than *Slc39a8* was differentially expressed. SLC30 (ZnT) zinc transporters move Zn^2+^ out of the cell, while ZIP8 moves Zn^2+^ into the cell, providing balance between intracellular and extracellular Zn^2+^ concentrations (reviewed in [32]). In the RNA-seq transcriptomics analysis [28], besides the expected *Slc39a8* downregulation in *Slc39a8*(*neo*/*neo*) mice, *Slc30a10* (the only one of ten *Slc30* family members) was upregulated in yolk sac, and downregulated in kidney and lung. From the point-of-view of survival, this observation in yolk sac would seem to make no sense: with SLC39A8 deficiency resulting in less intracellular Zn—combined with SLC30A10-mediated enhancement of intracellular Zn removal—the result would be catastrophic intracellular Zn depletion (and probably also Mn, Fe, Co, Se)!

Interestingly, many other differentially expressed channel genes (e.g., Ca^2+^ and Na^+^) were also found to be perturbed in *Slc39a8*(*neo*/*neo*) mice [28]. These findings suggest that the genome somehow “senses” the disappearance of “normal” ZIP8 function in these knockdown mice—thereby “deciding” which other transporter genes “need to be tweaked” as a mechanism for the best chances of survival.

How does this happen? The “genetic compensation response” is currently the best explanation for gene-expression differences between gene-knockout or gene-knockdown vs wild-type animals [33, 34]. Using zebrafish knockdown and knockout models [35], it was discovered that particular mRNAs carry a premature termination codon—which promptly triggers a *genetic compensation response* involving UPF3A (member of the nonsense-mediated mRNA decay pathway) and components of the COMPASS complex, i.e., enhancement of histone H3 Lys4 trimethylation (H3K4me3) at transcription start-site regions of compensatory genes; this was not found in “neutral” genes. Transcriptomics analysis of those alleles displaying mutant mRNA decay revealed upregulation of a substantial proportion of genes—in the gene group that exhibits sequence similarity to the mutated gene’s mRNA [36]—which is also consistent with the likelihood that the *genetic compensation response* involves a sequence-dependent mRNA mechanism.

These data [33–36] therefore suggest *SLC39A8* mRNA might carry a “recognition sequence” (i.e., a number of contiguous nucleotides) that provides a message for the coordinated up- or downregulation of *SLC* mRNAs and mRNAs of other differentially-expressed Ca^2+^ and Na^+^ channel genes seen in the transcriptomics study [28]. Future experiments to prove or disprove this hypothesis can be performed simply by bioinformatics analyses, comparing relevant mRNAs with “neutral gene” mRNAs.

The human genome contains 49 *ABC* genes in eight subfamilies (https://www.genenames.org/ and reviewed in [37]). The A2780 human ovarian cancer cell is a source for cisplatin- and adriamycin-resistant cell sublines; curiously, mRNA expression of seven *ABC* genes was increased and three *ABC* genes decreased. Expression of 32 *SLC* genes was also altered—17 increased and 15 decreased; *SLC39A8* was among five *SLC* genes upregulated > 10-fold [38]. This phenomenon of “drug-transporter gene expression readjustment, in response to cisplatin or adriamycin” appears to be another example of the *genetic compensation response* [35, 36], as discussed above for the *Slc39a8*(*neo*/*neo*) mouse [28].

To understand why ZIP8 deficiency in *Slc39a8*(*neo*/*neo*) mice results in the up- or downregulation of so many other transporter genes [28]—or why cisplatin or adriamycin resistance in A2780 cells causes dysregulation of ten *ABC* genes and 32 *SLC* genes—are fascinating observations for future experiments.

### SLC39A8 participation in fundamental cell processes

ZIP8 provides the cell with at least five essential trace elements (e.g., Mn, Zn, Fe, Se, Co)—which, in turn, likely feed signals into many downstream pathways (vide supra). ZIP8-associated pathways were therefore explored in various “ZIP8-activity gain” vs “ZIP8-activity loss” cell culture systems, in addition to the above-described mouse models. These studies have led to an appreciation that ZIP8 is involved in fundamental cell processes that include cell morphology, adhesion, migration, and cell proliferation.

For example, participation of ZIP8 downstream targets was investigated in *Slc39a8*-overexpressing *BTZIP8*-*3* lung, and in *Slc39a8* up-regulated and *Slc39a8* down-regulated cell culture model systems [39]. Interestingly, in *BTZIP8*-*3* mice (exhibiting ~2.5 times higher ZIP8 expression), lung showed re-organization of filamentous actin (F-actin)—especially enriched around branches of the trachea. ZIP8 overexpression in cultured mouse embryonic fibroblast (MEFs) was accompanied by substantial morphological changes and F-actin re-organization, as well as enhanced rates of cell proliferation and cell migration [39]. In *SLC39A8*-knockout HAP1 cells (a near-haploid cell line derived from human chronic myelogenous leukemia), morphological changes were consistent with increased cell-cell adhesion [39].

NFκB is a *protein complex* that participates in many cellular responses to stimuli—as diverse as oxidative stress, cytokines, free radicals, ultraviolet irradiation, oxidized LDL, and bacterial or viral infections. SNAIL2 is a transcriptional repressor encoded by the *SNAI2* gene. NFκB and SNAIL2 were elevated in *Slc39a8* upregulated MEFs and lung of the *BTZIP8*-*3* mouse, and decreased in *SLC39A8* downregulated HAP1 cells [39]. Expression levels of collagen type-I α2 chain (COL1A2) and E-cadherin (CDH1)—two downstream targets of NFκB and SNAIL2—also paralleled ZIP8 expression levels [39]. These data provide further evidence that fundamental functions of *SLC39A8*-encoded ZIP8 likely involve participation in cell morphology and cytoskeleton formation; these findings are not surprising, given that *SLC39A8* gene expression is known to occur in pluripotent ES cells [25].

Monocytes recruited to inflamed arteries, which then adhere to blood vessel walls, are essential for development of atherosclerosis. Because Zn homeostasis is known to participate in monocyte adhesion and recruitment, expression levels of mouse Zn transporters in “non-adhering” vs “adhering” monocytes were compared. After screening expression levels of all 14 *Slc39a*-encoding Zn importers and all ten *Slc30a*-encoding Zn efflux transporters—Zn-dependent *Slc39a8* was shown to be the only transporter upregulated in monocytes that adhered to aorta ex vivo [40]; however, this increase was only 2-fold. Although *Slc39a8* overexpression was demonstrated to increase uptake of Zn, Fe, and Cd in monocytes, only Zn supplementation of endothelial monolayers in cell culture was confirmed to be accountable for enhancing adhesion of monocytes to endothelial cells. In *Apoe*(*−*/*−*) knockout mice fed a “Western high-fat diet,” Zn-dependent *Slc39a8* upregulation was even more strongly associated with increased monocyte adhesion and recruitment to nascent atherosclerotic lesions [40].

SLC39A8 was also discovered to be involved in the cell’s response to the anti-cancer drug, cisplatin. ZIP8 overexpression in MEFs was found to increase cisplatin sensitivity, whereas ZIP8-knockout HAP1 cells displayed cisplatin resistance; in these two cell lines and the *BTZIP8*-*3* mouse, cisplatin was established not to be a ZIP8 transporter substrate [41]. Moreover, in MEFs and in the *BTZIP8*-*3* mouse, ZIP8-overexpression was shown to be correlated with decreases in the anti-apoptotic protein BCL2, whereas in ZIP8-knockout HAP1 cells and in the *Slc39a8*(*neo*/*neo*) mouse, increased BCL2 expression was seen. ZIP8 overexpression was also associated with cisplatin-induced apoptosis—as confirmed by an elevation in cleaved CASPASE 3 protein [41]. These data further underscore the ubiquitous functions and participation of the SLC39A8 transporter in innumerable fundamental cell processes.

## SLC39A8 Clinical Studies

### Human *SLC39A8* and the immune system

The *SLC39A8* gene was first stumbled upon in human monocytes that had been stimulated with either *Mycobacterium bovis* BCG cell wall or lipopolysaccharide (LPS), but was given the obscure name “BIGM103”; when a cDNA library—prepared from monocytes stimulated with *M*. *bovis* BCG cell wall—was screened [42], a novel transcript was found to be upregulated by the inflammatory cytokine, tumor necrosis factor (TNF). Expression of this transcript was negligible in unstimulated monocytes, whereas elevated expression levels of transcript were seen during differentiation of monocytes to dendritic cells or macrophages. The transcript’s open reading frame encoded a putative transmembrane protein showing homology with several proteins in the database that were functionally unknown at that time, but authors noted that the protein had substantial similarity to the “ZIP family of metal transporters,” as well as possessing the hallmark of Zn-metalloproteases [42].

SLC39A8 function was then shown in human lung to protect against inflammation [43]. Focusing on the role of Zn as an essential micronutrient and cytoprotectant regarding host response to inflammatory stress, authors quantified mRNA transcripts of two dozen Zn transporters—the 14 known *SLC39* importers and ten known *SLC30* exporters (https://www.genenames.org/). Studies in primary lung epithelial cells obtained from human donors and in BEAS-2B (human polyomavirus-transformed bronchus epithelial) cell cultures were carried out; TNF-treated vs untreated cells were compared and, of the 24 transcripts examined, only *SLC39A8* mRNA was markedly induced by TNF [43]. Increased *SLC39A8* expression was associated with elevated intracellular Zn content, and this coincided with successful cell survival when TNF was present. Authors concluded that upregulation of human SLC39A8, by functioning as an essential zinc uptake transporter early in the inflammatory process, is sufficient to protect lung epithelial cells against TNF-induced cytotoxicity [43].

Next, the mechanism by which Zn appears to regulate NFκB activity during innate immune activation was investigated. As mentioned earlier, the transcriptional factor NFκB represents a *protein complex* found in almost all cell types, participating in numerous responses to external stimuli. Intriguingly, the *SLC39A8* and *NFKB1* genes are located adjacent to one another on Chr 4q24; reciprocal regulation between two adjacent genes is known to occur in various organisms, indicating that coordinated expressional mechanisms are possible.

In cell culture, the *SLC39A8* gene was shown to be initially activated by the transcription factor, NFKB1; this causes enhanced influx of Zn into monocytes and macrophages, leading to the coordinated NFKB1-mediated transcription of other inflammatory factor genes. The Chr 4 g.102532378C>T *NFKB1* intronic variant is an expression quantitative trait locus (eQTL) affecting the neighboring *SLC39A8* gene, and this eQTL appears to cause decreased *SLC39A8* mRNA expression in monocytes and macrophages [44]. Reciprocally, the ZIP8-mediated higher Zn levels stimulate *NFKB1* gene transcription, functioning negatively to regulate pro-inflammatory responses by means of Zn-mediated downregulation of IκB kinase (IKK) activity [45]. Moreover, *Slc39a8*(*neo*/*neo*) fetal fibroblasts exhibited decreased Zn uptake and increased NFκB activation; consistent with this finding, mice fed a Zn-deficient diet showed disproportionate inflammation caused by polymicrobial sepsis—concomitant with loss of normal IKK regulation [45]. These data thus identify a negative feedback loop involving *SLC39A8* that directly controls innate immune function through coordination of Zn metabolism and *NFKB1* gene transcription.

Following LPS-induced inflammation in human macrophages, extracellular Zn dramatically decreases interleukin-10 (IL10) mRNA expression and IL10 protein release; in contrast, *TNF*, *IL8*, and *IL6* transcripts are increased [45]. *SLC39A8* knockdown inhibits LPS-driven cellular accumulation of Zn, also preventing the Zn-dependent reduction of IL10 release. Furthermore, Zn supplementation in culture medium decrease nuclear localization and activity of C/EBPβ, a transcription factor known to drive *IL10* expression. It was concluded that Zn regulates LPS-mediated immune activation of human macrophages in a ZIP8-dependent manner, as well as lowering IL10 levels; these findings suggest Zn-mediated homeostasis in macrophages plays a pivotal role in host defense against pathogens [45].

Phytohemagglutinin (PHA), which causes potent mitogen-inducing activation and proliferation of lymphocytes, was used to stimulate T cells in culture; from human subjects who had received oral Zn supplementation (15 mg/day), T cells were collected and grown in culture [18]. Compared to volunteers not receiving oral Zn, those on Zn supplementation showed higher expression of PHA-activated interferon-γ (IFNG)—indicating that Zn potentiates T cell activation. Similarly, Zn treatment of PHA-activated T cell cultures resulted in increased *IFNG* expression. When *SLC39A8* mRNA was knocked-down by siRNA, decreased ZIP8 levels resulted in less T cell activation; transiently transfected *ZIP8* overexpression led to enhanced T cell activation. These findings indicate that, along with the role in human monocytes and macrophages, ZIP8 also participates in Zn-mediated T cell activation [18].

### *SLC39A8*, Mn-deficient glycosylation defect, and dysmorphogenesis

Chronologically, after studies by the Knoell lab had begun—concerning the importance of SLC39A8 in human lung to protect against inflammation and cytotoxicity [43]—genome-wide association studies (GWAS) began to appear, reporting correlations between a *SLC39A8* genetic variant and various clinical disorders (Table 1). In all cases, these mutant alleles caused diminished ZIP8 function. Just as with the mouse studies, the number of organs, systems, and cell types affected by deficient ZIP8 expression has become staggering (Table 1).

**Table 1:** *SLC39A8* allelic variants found to be associated with clinical disorders

cDNA	Protein	Phenotype	Reference(s)
c.97G > A	p.Val33Met	(?)Dysmorphogenesis; Mn-deficient hypoglycosylation	[17]
c.112G > C	p.Gly38Arg	Dysmorphogenesis; Mn-deficient hypoglycosylation	[17, 47]
c.338G > C	p.Cys113Ser	Dysmorphogenesis; Mn-deficient hypoglycosylation; Leigh-like mitochondrial disease	[20]
c.610G > T	p.Gly204Cys	Dysmorphogenesis; hypoglycosylation	[17]
c.1004G > C	p.Ser335Thr	(?)Dysmorphogenesis; hypoglycosylation	[17]
c.1019 T > A	p.Ile340Asn	Dysmorphogenesis; hypoglycosylation	[17]
c.1172C > T	p.Ala391Thr	Lower serum HDL-Chol levels	[48–50]
		Increased risk of coronary artery disease	[51]
		Increased body mass index (BMI)	[52, 53]
		Increased risk of (systolic & diastolic) hypotension	[54]
		Increased risk of dilated cardiomyopathy	[55]
		Smoking-induced atherosclerotic plaques	[56]
		Elevated NT-proBNP levels	[57]
		Increased risk of acute coronary syndrome	[57]
		Increased risk of cardiovascular death	[57]
		Increased risk of liver inflammation and fibrosis	[58]
		Increased bronchodilator response to albuterol	[44]
		Increased plasma VWF levels, risk of ischemic stroke	[59]
		Increased risk of schizophrenia	[50, 60, 61]
		Increased risk of Parkinson disease	[50]
		Increased risk of Crohn disease	[50, 62]
		Increased risk of myopia	[50]
		Increased risk of allergy	[50]
		Decreased height	[50, 53]
		Increased risk of inflammatory bowel disease	[50]
		Increased risk of cerebrovascular disease	[63]
		Increased risk of adolescent idiopathic scoliosis	[53]
		Increased risk of SLE-primary-Sjögren syndrome	[64]
microRNA 488 targeting of *SLC39A8* mRNA		Inadvertent participation in the inflammatory progression of OA	[65]

The two question marks “(?)” denote variants seen in one patient who had two *SLC39A8* mutations on one chromosome; thus, until these individual amino acid changes are tested independently, it remains unknown which mutation(s) is(are) responsible for the hypomanganesemia and other observed pleiotropic effects in that patient (see text for details). *NT*-*proBNP* N-terminal pro-B-type natriuretic peptide, *VWF* von Willebrand factor, *SLE* systemic lupus erythematosus, *OA* osteoarthritis

An autosomal recessive pattern of developmental abnormalities was recognized in six individuals from a Hutterite community in Canada, as well as in a sibling pair from an Egyptian family; the disorder was characterized by mental retardation, developmental delay, hypotonia, strabismus, cerebellar atrophy, and variable short stature [47]. Whole-exome sequencing of affected individuals identified the same *SLC39A8* homozygous variant—c.112G>C (p.Gly38Arg). The afflicted Hutterite and Egyptian individuals did not share an extended common haplotype, indicating that this mutation must have arisen independently. The eight affected individuals exhibited variably low levels of Mn and Zn in blood, and elevated Mn and Zn levels in urine, consistent with renal wasting [47].

In an independent study, whole-exome sequencing was carried out in a German child presenting with cranial asymmetry, severe infantile spasms with hypsarrhythmia, and disproportionate dwarfism. Authors noted that transferrin glycosylation was strikingly diminished—suggesting type II congenital disorder of glycosylation (CDG); in addition, blood Mn levels were extremely low [17]. Two *SLC39A8* variants were found in this patient—c.112G>C (p.Gly38Arg) and c.1019T>A (p.Ile340Asn). Among a group of unresolved patients diagnosed with CDG, another individual was then discovered; this patient carried *SLC39A8* variants c.97G>A (p.Val33Met) and c.1004G>C (p.Ser335Thr) on the paternal allele, and c.610G>T (p.Gly204Cys) on the maternal allele (Table 1).

Patients with these *SLC39A8* variants [17, 47] showed impairment of Mn-dependent enzyme activities—most notably β-1,4-galactosyltransferase, a Golgi enzyme essential for biosynthesis of the carbohydrate portion of glycoproteins [17]; it should be emphasized that about half of all translated proteins in eukaryotes are posttranslationally *N*-glycosylated [66]. Impaired galactosylation is known to result in severe disorders with deformed skull, severe seizures, short limbs, profound psychomotor retardation, and hearing loss.

Oral galactose supplementation was successful in normalizing glycosylation function in the two German patients [17]. A subsequent report by the German group confirmed that high-dose Mn therapy is also effective in reversing impaired galactosylation in the two SLC39A8-deficient patients; however, careful monitoring (i.e., glycosylation assays and blood Mn measurements) is required in order to prevent Mn toxicity [67].

In siblings born to consanguineous Lebanese parents, an additional *SLC39A8* deficiency was reported; two sisters exhibited profound developmental delay, dystonia, seizures, failure to thrive, and features of Leigh-like mitochondrial disease [20]. Brain magnetic resonance imaging of both siblings identified bilateral basal ganglia hyperintensities and cerebral atrophy. Mitochondrial respiratory-chain studies were performed only for patient 1, and this revealed lowered complex IV and II **+** III activity in liver, combined with elevated complex I activity; in muscle of patient 1, complex IV activity was borderline low, and pyruvate dehydrogenase activity was decreased [20]. Whole-genome sequencing found a new *SLC39A8* variant—g.103236869C>G; c.338G>C; p.Cys113Ser. Mn levels in patient 2 blood and urine were undetectable, and transferrin electrophoresis of patient 2 serum confirmed a type II CDG defect [20]. This study thus extended the previous reports [17, 47] by discovering yet-another *SLC39A8* variant that, when homozygous, causes type II CDG; moreover, this report suggests that deficient ZIP8 in mitochondria can cause a Leigh-like syndrome—perhaps associated with diminished activity of Mn-dependent enzymes such as β-galactosyltransferase and/or mitochondrial manganese-superoxide dismutase (MnSOD) [20].

To determine the function of *SLC39A8* mutants associated with CDG and Leigh syndrome, four mutant alleles were constructed and transfected into HeLa cells, and the results were compared with the consensus (wild-type) *SLC39A8* cDNA; the selected *SLC39A8* mutants included Gly38Arg, Gly38Arg **+** Ile340Asn, Val33Met **+** Gly204Cys **+** Ser335Thr, and Cys113Ser [19]. Whereas consensus *SLC39A8* increased ^54^Mn uptake in wild-type cells, all four selected alleles lacked ZIP8-mediated Mn uptake into the cells—thereby providing an explanation for the severe Mn deficiency seen in those CDG and Leigh syndrome patients. It is noteworthy that no differences in Zn, Fe, or Cu uptake were observed between the consensus and the four mutant *SLC39A8* cell lines. All four mutants also failed to localize the SLC39A8 protein on the cell surface; instead, the SLC39A8 protein was retained within the endoplasmic reticulum. Interestingly, ^54^Mn levels in mitochondria and MnSOD activity were decreased in the mutant cell lines, resulting in enhanced oxidative stress [19].

These data underscore the importance of normal *SLC39A8* expression in preventing CDG and Leigh syndrome, and in mediating Mn uptake and mitochondrial function [19]. It is unfortunate that each of the mutated amino acids was not studied individually; hence, Table 1 includes two question marks for those variants in which it remains unclear whether that particular amino acid change was responsible for defective Mn uptake—versus being a “silent passenger” mutation and not the one causing Mn-deficient hypoglycosylation. Note that all six of these SNVs differ from the c.1172C>T; p.Ala391Thr variant that will be described in all other clinical studies (vide infra).

### *SLC39A8* and the cardiovascular system

The first GWAS to report a *SLC39A8* variant appeared in a meta-data analysis of 15 combined studies, comprising >55,000 participants; moreover, authors screened for correlations between SNVs at “lipid-related” loci and risk of coronary artery disease in ~9600 cases and ~38,600 controls [48]. Among four novel genetic loci—showing reproducible statistically significant associations with lipids—was a *SLC39A8* SNV (rs13107325; c.1172C>T transition; p.Ala391Thr; minor allele frequency (MAF) = 0.08; *P* = 1.6 × 10^−8^) that was correlated with HDL-Chol levels (Table 1); the amino acid change of Ala-391 to Thr-391 is associated with lower *SLC39A8* expression levels [48].

In the same year, looking for common variants associated with plasma lipids in ~99,900 individuals of European ancestry, a GWAS reported 95 significantly associated loci (*P* < 5.0 × 10^−8^), 59 of which demonstrated genome-wide significant associations with lipid traits; the same *SLC39A8* minor allele (p.Ala391Thr; MAF = 0.07) was significantly correlated (*P* = 7.0 × 10^−11^) not only with serum-circulating HDL-Chol levels but also with coronary artery disease [51].

Body mass index (BMI) was assessed in GWAS of 123,900 individuals, with targeted follow-up of 42 SNVs in ~125,900 additional individuals; 14 known obesity-susceptibility loci, plus 18 new loci, were associated with increased BMI, one of which included the *SLC39A8* p.Ala391Thr variant (*P* < 1.5 × 10^−13^) [52]. Another GWAS screened for the traits of low-density lipoprotein cholesterol (LDL-Chol), HDL-Chol, triglycerides, and total cholesterol; >188,500 individuals were examined, and 157 statistically significant (*P* < 5.0 × 10^−8^) loci having correlations with lipid levels were identified [49]. Using dense genotyping in individuals of European, East Asian, South Asian, and African ancestry—authors narrowed the association signals to 12 loci, one of which was the *SLC39A8* p.Ala391Thr variant that was again highly associated (*P* < 1.1 × 10^−15^) with HDL-Chol [49]. It is worth noting that this p.Ala391Thr variant was found in subjects only of European ancestry, but is virtually absent in those from the other ethnic groups.

Similar to the cell culture studies with four *SLC39A8* mutants described above [19], the consensus ZIP8 Ala-391 wild-type variant was compared with the Thr-391 variant in human embryonic kidney HEK293 cell culture [68]. Following incubation with Cd, the Thr-391 variant was found to have lower intracellular Cd levels with accompanying less Cd-induced toxicity, decreased phosphorylation of mitogen-activated protein kinase-1 (MAPK1), and lowered NFκB activation; not surprisingly, the same differences were seen in vascular endothelial cells [68]; although the authors suggest that the ZIP8 Thr-391 variant is “therefore mechanistically responsible for lower serum HDL-Chol levels, coronary artery disease, and hypotension”—this connection remains to be elucidated in their study.

To understand genetic architecture of blood pressure and to assess effects on target organ damage, a GWAS was performed from targeted and genome-wide arrays in >201,500 individuals of European ancestry, plus genotypes of an additional >140,800 individuals for validation; authors identified 66 blood pressure-associated loci, of which 17 were new, and 15 harbored pleiotropic distinct association signals [54]. There were 66 index SNVs enriched for *cis*-regulatory elements—particularly in vascular endothelial cells—consistent with a primary role in blood pressure control through modulation of vascular tone across multiple tissues; the combination of these 66 index SNVs in a risk score showed comparable effects in >64,400 additional individuals. The same *SLC39A8* variant (p.Ala391Thr) was significantly associated with both reduced systolic (*P* = 3.3 × 10^−14^) and diastolic (*P* = 2.3 × 10^−17^) blood pressure [54].

Dilated cardiomyopathy (DCM) is a substantial cause of heart failure with a strong hereditary component. A whole-exome-wide array-based association study included ~2790 DCM patients and ~6870 control subjects from six populations of European ancestry. In addition to two previously identified associations with SNVs, six novel DCM-associated loci, including the *SLC39A8* Ala391Thr variant (*P* = 6 × 10^−7^), were identified. All eight candidate genes—except *SLC39A8*—that contribute to sporadic DCM, exhibited preferential expression in cardiac striated muscle [55].

Smoking is a risk factor for atherosclerosis, with well-known effects on gene expression in circulating blood cells. In order to study genome-wide expression profiles and totals of atherosclerotic plaques in carotid arteries, authors collected circulating monocytes from 248 smokers and 688 non-smokers from French subjects; patterns of co-expressed genes were identified by independent component analysis (ICA), and a likelihood-based causality test was implemented to select patterns that fit models containing the path “smoking → gene expression → plaques” [56]. The network that exhibited the strongest support for causal effect associated with plaques was discovered to be *SLC39A8*; this is a credible candidate because of known correlations with HDL-Chol [48, 49]—as well as cellular uptake of Cd [12], a metal that is abundantly present in tobacco [69]. Analysis of the transcriptome in monocytes revealed candidate genes that could easily have been missed by expression-phenotype association analysis alone. Note that this study in human monocytes [56] is consistent with the earlier findings reported in mouse Zn-deficient monocytes that exhibit enhanced adhesion to aorta ex vivo [40] [vide supra].

Natriuretic peptides are secreted by cardiomyocytes in response to cardiac stretch, as happens during heart failure; NH_2_-terminal pro-B-type natriuretic peptide (NT-proBNP) is a strong predictor of mortality in coronary artery disease and is widely employed as a prognostic indicator. Out of >18,600 enrolled patients with acute coronary syndrome, a GWAS and Mendelian randomization study of NT-proBNP was carried out with ~3740 patients—plus an additional set of ~5490 patients from the same trial, used for validation [57]. The same above-mentioned deleterious allele of *SLC39A8* (p.Ala391Thr) was statistically significantly associated (pooled *P* = 6.0 × 10^−10^) with increased NT-proBNP levels. This *SLC39A8* variant was also correlated with higher risk of cardiovascular death (HR = 1.39, 95% CI 1.08–1.79, *P* = 0.0095), which in this study was the only variant associated with a clinical outcome [57].

### *SLC39A8* and liver

Whereas lowered serum HDL-Chol levels [48–50] and increased BMI [52, 53] are described earlier (in the “cardiovascular system” section), liver metabolism clearly plays a substantial role in these phenotypes. The same holds true for Mn-deficient hypoglycosylation [17, 20, 47] and the Leigh syndrome-like mitochondrial redox deficiency [20] (vide supra). To what extent any of these traits, or any of the other *SLC39A8* variant-associated phenotypes (Table 1)—includes a hepatic SLC39A8-mediated contribution—remains to be determined.

Non-alcoholic fatty liver disease (NAFLD) can lead to liver inflammation and subsequent fibrosis (non-alcoholic steatohepatitis, NASH). The etiology of NAFLD and NASH is complex—including dietary differences, immunity, inflammation, microbiome composition, and alterations in metabolic traits. A GWAS of hepatic inflammation and fibrosis markers in a large clinical cohort would be extremely difficult, because liver biopsy is an invasive procedure with significant risks; however, employing non-invasive corrected T1-magnetic resonance imaging (cT1-MRI) would be one solution to the problem. Increased nuclear magnetic resonance T1 relaxation times in extracellular fluid are consistent with fibrosis and inflammation. Using data from UK Biobank and principal component analysis, authors generated a discovery cohort of ~2290 Caucasian British individuals, followed by an independent replication cohort of 212 European non-Caucasian individuals from UK Biobank; intriguingly, the one SNV associated with liver cT1-MRI findings that reached statistically high significance (*P* = 3.4 × 10^−32^) was the *SLC39A8* p.Ala391Thr variant (Parisinos CA, Wilman HR, Thomas EL, Hemingway H, Banerjee R, Yaghootkar G, manuscript submitted [58]).

In a recent mouse study, hepatic ZIP8 deficiency was associated with Se dysregulation, liver inflammation and fibrosis, and neoplastic changes—consistent with hepatocellular carcinoma [70]. The role of NFκB in liver is crucial, underlined by the fact that genetic ablation of regulators of NFκB in mouse models leads to spontaneous liver injury, fibrosis, and hepatocellular carcinoma [71]. Keeping in mind that mice receiving a Zn-deficient diet develop disproportionate inflammation in response to polymicrobial sepsis—along with NFκB activation and loss of normal IKK regulation [45]—these data indicate that ZIP8 participates in a negative feedback loop directly involved in regulation of innate immune function via coordinated Zn metabolism [45]. Consequently, the *SLC39A8* p.Ala391Thr variant, discovered in the liver cT1-MRI study [58], which is correlated with decreased *SLC39A8* expression in liver, is likely to be correlated with stimulation of the NFκB pathway. Therefore, discovery of this *SLC39A8* variant associated with cT1-MRI detection of liver inflammation and fibrosis markers [58] would seem to be a credible candidate involved in the clinical disorder, NASH.

Hepatic zinc deficiency is a well-documented finding in alcoholic patients. After 5 months of ethanol vs control diet in rats, Zn levels were shown to be substantially decreased in liver endoplasmic reticulum and mitochondria; mitochondrial ZIP8, ZIP13, and the Zn exporter SLC30A4 (ZnT4) levels were increased—along with enhancement of C/EBPβ, cytochrome *c* release, CASPASE 3 activation, and apoptotic cell death [72]. In a GWAS of alcohol use in ~480,000 subjects of European descent to decipher the genetic architecture of alcohol intake (https://www.biorxiv.org/content/biorxiv/early/2018/10/30/453332.full.pdf), authors identified 46 novel loci (which included the *SLC39A8* Ala391Thr variant), and investigated their potential functional significance using MRI, gene expression, and behavioral studies in *Drosophila*; the newly identified genetic pathways associated with alcohol consumption suggested common genetic interactions with several neuropsychiatric disorders including schizophrenia.

### Conditional cell type-specific *Slc39a8* knockout studies

Although *Slc39a8(−/−)* global knockout mice are early-embryolethal, *Slc39a8* conditional knockout mice have been constructed and shown to be viable. This approach allows for exploration of ZIP8 functions in later developmental stages, e.g., in cardiomyocytes and hepatocytes.

A *UBC>Cre>ERT2>Slc39a8*(*fl*/*fl*) (“*Slc39a8*-inducible global-knockout”) viable mouse was therefore generated, in which *Slc39a8* ablation can be triggered by tamoxifen treatment at any age; an *Alb>Cre>Slc39a8*(*fl*/*fl*) (hepatocyte-specific *Slc39a8* knockout) was also constructed [73]. Dramatically decreased Mn levels were observed in multiple organs and in whole blood of both mouse models, compared with controls, whereas neither transgenic mouse line exhibited any significant differences in high-density lipoprotein-cholesterol (HDL-Chol), body weight, or overt neurological or skeletal abnormalities [73]. In order to test whether human *SLC39A8* could compensate for absence of mouse *Slc39a8*, an AAV-vector expressing human *SLC39A8*—under control of a liver-specific promoter—was injected into the *Alb>Cre>Slc39a8*(*fl*/*fl*) mouse; human *SLC39A8* expression in liver restored Mn levels in liver and kidney. The liver-specific *Slc39a8* knockout also showed decreased liver and kidney activity of the Mn-dependent enzyme arginase. Both mouse models demonstrated deficient protein *N*-glycosylation. It was concluded that normal levels of hepatic ZIP8 reclaim Mn from bile, thereby regulating whole-body Mn homeostasis, which in turn normalizes activity of all Mn-dependent enzymes [73].

While attempting to characterize the *UBC>Cre>ERT2>Slc39a8*(*fl*/*fl*) *Slc39a8(−/−)* global knockout [74], it was discovered that before early-embryonic death, the mice show a cardiac phenotype similar to human left ventricular noncompaction (LVNC). Because SLC39A8 has been implicated in extracellular matrix (ECM) degradation [75], which would be consistent with a LVNC-type of defect, heart muscle of a myocardial-specific *Slc39a8* knockout was studied**;** myocardiocytes showed striking ECM accumulation and decreases in several ADAMTS-metalloproteinases [74]. Consistent with the intact animal observations, knockdown of *SLC39A8* in normal human umbilical vein endothelial cells (HUVECs) in culture, blocked *ADAMTS1* transcription by decreasing cellular Zn uptake and, consequently, diminished metal regulatory transcription factor-1 (MTF1) transcriptional activity. Clinically, isolated LVNC is the result of excessive trabeculation and impaired myocardial compaction during heart development; the ECM, which separates endocardium from myocardium, plays a critical role in ventricular trabeculation and compaction. These data therefore identify SLC39A8 as an important player underlying the development of ventricular trabeculation and compaction, as well as participating in an ECM-regulatory pathway during myocardial morphogenesis [74].

### *SLC39A8* and kidney

In patients with chronic kidney disease (CKD), cardiovascular disorders are prevalent and responsible for approximately half of all CKD-related deaths. Cardiac biomarkers are important in accurate diagnosis and prompt management of heart failure and acute coronary syndrome; there is increased awareness of novel cardiac indicators that may improve diagnostic accuracy reflecting myocardial injury, inflammation, and remodeling. Interpretation of these biomarkers can be complicated, because elevated levels may not reflect myocardial injury or heart muscle tension—but rather might reflect decreased urinary clearance with retention of solutes and/or overall CKD-associated chronic inflammation. Emerging cardiac indicators include NT-proBNP, produced by cardiomyocytes but also by kidney [reviewed in [76]].

It was noted earlier that the *SLC39A8* (p.Ala391Thr) allele was highly significantly associated with NT-proBNP levels [57]. In the transcriptomics analysis of the *Slc39a8*(*neo*/*neo*) knockdown mouse [28], kidney exhibited highly significant upregulation of *Npr3* (natriuretic peptide receptor-3). In a *Sglt2>Cre>Slc39a8*(*flox*/*neo*) conditional knockout in which renal epithelial *Slc39a8* expression was ablated, atrial natriuretic peptide (ANP) levels were markedly decreased (Jorge-Nebert L, Soleimani M, and Nebert DW, unpublished). ANPs are known to dilate blood vessels and induce natriuresis and diuresis—resulting in lowered blood pressure and blood volume; in part, ANPs counterbalance actions of the renin-angiotensin-aldosterone and neurohormonal systems, thereby playing a pivotal role in cardiovascular regulation [77]. In *Slc39a8*(*neo*/*neo*) liver, angiotensin-1-converting enzyme-2 (*Ace2*) was also upregulated [28], perhaps helping to explain the potential clinical role of *SLC39A8* in heart disease. If SLC39A8 deficiency causes ANP depletion, it seems plausible that upregulation of the renal NPR3 receptor might follow. In conclusion, SLC39A8-associated kidney function is intimately interconnected with cardiac disease.

### *SLC39A8* and lung

In a GWAS pharmacogenomics study of ~1440 asthmatic children [44]—selected from the two tails of extreme phenotypes of “bronchodilator drug response to albuterol”—statistically suggestive (*P* < 7.06 × 10^−6^) loci were found located near genes previously associated with lung capacity (*DNAH5*), immunity (*NFKB1* and *PLCB1*), and beta-adrenergic signaling (*ADAMTS3* and *COX18*). Analysis of the bronchodilator-drug-response-associated variant in *NFKB1* revealed a potential regulatory function in bronchial smooth muscle cells [44]. Given the relevance of NFκB in immune pathways and asthma, genomic-sequencing experiments were performed to identify intronic *NFKB1* SNVs that might regulate expression of neighboring genes; among genes within 1 Mb of the *NFKB1* gene as a reliable cutoff, the low bronchodilator-response-associated T allele of the Chr 4 g.102532378C>T *NFKB1* intronic variant was found to be significantly associated with decreased *SLC39A8* mRNA expression in white blood cells (*P* = 0.0066, FDR-adjusted *P* = 0.0856, log_2_(β) = − 0.327) [44]. This finding was also noted in the “Immune System” section (vide supra).

### SLC39A8 and the coagulation system

Meta-analysis of GWAS data from >46,300 individuals of European, African, East Asian, and Hispanic ancestry was carried out to identify, and functionally test, novel genetic associations regulating the coagulation factor-8 (FVIII) and its carrier protein von Willebrand factor (VWF) plasma levels, with risk of arterial and venous thrombosis. Beyond the ten previously reported associations with these phenotypes, 13 novel genome-wide significant (*P* ≤ 2.5 × 10^−8^) associations—seven with FVIII levels and 11 with VWF levels—were identified; interestingly, the rs6855246 SNV located near the *SLC39A8* Ala391Thr variant, correlated with increased VWF levels (*P* = 8.68 *×* 10^−10^), was found, but only in the European cohort of >42,000 individuals [59]. Further, this linkage-equilibrium correlation was confirmed experimentally by silencing *SLC39A8* mRNA expression in culture, which enhanced VWF release into the medium. These findings suggest that SLC39A8-mediated metal ion uptake participates in regulation of plasma VWF levels on ischemic stroke risk; whether this involves Mn, Zn, Fe, Se, and/or Co—remains to be determined.

### *SLC39A8* and the central nervous system

Another early GWAS discovery of a *SLC39A8* variant involved a case-control study of 476 schizophrenia patients and 447 control subjects from Galicia, combined with a replication sample comprising >4000 cases and >15,100 control subjects of European origin**;** the SNV (rs13107325; p.Ala391Thr) was somewhat significant (*P* = 2.7 × 10^−6^) in the collective sample, following Bonferroni correction [60]. Possible etiology—as to why deficient metal cation uptake in the central nervous system (CNS) might be correlated with schizophrenia—is not understood.

Discovery of a *SLC39A8* variant allele with schizophrenia was quickly followed up by a considerably larger GWAS of >36,900 cases and >113,000 controls; among 108 highly statistically significant loci identified, the above-described *SLC39A8* (p.Ala391Thr) gene variant (*P* = 8.0 × 10^−15^) was found [61], thereby confirming the original 2010 study [60]. Associations were enriched among genes expressed in the CNS, providing biological plausibility for their findings; independent of genes expressed in brain, associations were enriched among genes expressed in tissues that have important roles in immunity—providing support for a speculative link between the immune system and schizophrenia. Previous studies showing participation of ZIP8-mediated Zn uptake during inflammation and innate immune activation [43, 45, 46] combined with these GWAS showing a relationship between purported diminished ZIP8 function and CNS function [60, 61], suggest that *SLC39A8* expression is likely involved in the “brain-gut-microbiome” axis (reviewed in [78]).

Subsequently, a scan for genetic variants associated with multiple phenotypes, by comparing a very large GWAS of “42 traits or diseases,” identified 341 loci. Several loci were correlated with multiple phenotypes; for example, the *SLC39A8* p.Ala391Thr allele was shown to influence seven of the 42 traits [50]—including**:** increased risk of schizophrenia [log-transformed odds ratio (log OR) = 0.15; (*P* = 2.0 × 10^−12^)], Parkinson disease [log OR = − 0.15; (*P* = 1.6 × 10^−7^)], Crohn disease, myopia, and allergy; lower serum HDL-Chol levels; and decreased height (Table 1). Using these loci to identify phenotypes that have multiple genetic causes in common—is informative; for example, variants associated with increased risk of schizophrenia also tended to be associated with increased risk of inflammatory bowel disease [50].

Because deviation from normal adolescent brain development precedes manifestations of many major psychiatric symptoms, a one-group-at-a-time GWAS was performed in a cohort of healthy 14-year-old adolescents, followed by validation of the findings in four independent samples across the life span with allele-specific expression analysis of top “hits”; groups of identified gene-brain associations among patients with schizophrenia, unaffected siblings, and healthy control individuals were compared [79]. Gray matter volume was assessed by neuroimaging in a discovery sample of >1700 adolescents, and in a replication sample of ~8690 healthy adults. The *SLC39A8* Ala391Thr variant was associated with larger gray matter volume of the putamen, combined with decreased *SLC39A8* expression specifically in cells of the putamen (*P* = 1.7 × 10^−4^). The identified association was validated in samples across the life span—but was demonstrated to be significantly weakened in both patients with schizophrenia (*P* = .002) and unaffected siblings (*P* = .04). Thus, the *SLC39A8* missense mutation is correlated with larger gray matter volume in the putamen, but this association is significantly weakened in patients diagnosed with schizophrenia [79].

Moreover, an “unbiased phenome-wide approach” was used in an attempt to understand phenotypic implications of the association of the *SLC39A8* p.Ala391Thr variant with schizophrenia. In a large genomic biobank, 50 traits were generated—based on diagnostic codes using latent Dirichlet allocation, and these were examined for correlation with the risk variant; subsequently, any significant phenotypes were further characterized by examining any association with individual diagnostic codes contributing to the trait [63]. Among the 50 phenotypes, one was associated at an experiment-wide significance threshold (beta = 0.003; uncorrected *P* = 4.9 × 10^−4^), comprising predominantly brain-related codes—including “intracranial hemorrhage,” “cerebrovascular disease,” and “delirium/dementia” [63]. These findings suggest that the functional *SLC39A8* variant, previously associated with schizophrenia risk, is also correlated with increased liability to cerebrovascular disease.

Excessive alcohol consumption is associated with increased risk of schizophrenia. As mentioned earlier, a GWAS of alcohol use in ~480,000 people of European descent (https://www.biorxiv.org/content/biorxiv/early/2018/10/30/453332) identified 46 novel loci (including the SLC39A8 Ala391Thr variant)—which identified new genetic pathways associated with alcohol consumption and suggested common genetic mechanisms with several neuropsychiatric disorders comprising schizophrenia.

### *SLC39A8* and the musculoskeletal system

While attempting to understand osteoarthritis (OA) pathogenesis, authors examined expression profiles of miRNAs in chondrocytes derived from joint cartilage of OA patients, comparing those profiles with that from normal cartilage; the most potent miRNA and its target and functional role in OA pathogenesis were then investigated—using a target-validation system and a mouse model. Among those tested, microRNA 488 was most significantly decreased in OA chondrocytes [65]. In chondrocytes isolated from normal cartilage samples, IL1B treatment decreased, whereas TGFβ3 (TGFB3) treatment increased, microRNA 488 levels. Target-validation studies confirmed that microRNA 488 is able to target *SLC39A8* mRNA, and suppression of *Slc39a8* expression in the OA animal model decreased degradation of cartilage. It was thus suggested that microRNA 488 participates, in a beneficial way, during chondrocyte differentiation and cartilage genesis—by blocking *SLC39A8*-mediated upregulation of matrix metallopeptidase-13 (MMP13) activity that promotes OA [65].

In a subsequent related paper, authors studied participation of Zn homeostasis, Zn transporters, and Zn-dependent transcription factors during OA pathogenesis; among all Zn transporters in cartilage of both humans and mice afflicted with OA—increased *SLC39A8* expression was found to be associated with higher levels of intracellular Zn in diseased chondrocytes [75]. SLC39A8-mediated Zn influx results in upregulated expression of matrix-degrading enzymes (MMP3, MMP9, MMP12, MMP13, and ADAMTS5) in chondrocytes. Ectopic expression of *Slc39a8* in mouse cartilage tissue caused OA-related destruction of cartilage; in contrast, in chondrocyte-specific *Slc39a8(−/−)* knockout mice, surgically induced OA-related degradation of cartilage was suppressed, along with lower levels of Zn influx and the matrix-degrading enzymes. Moreover, MTF1 was discovered to be essential for regulating Zn-dependent ZIP8-mediated catabolism, and genetic downregulation of *Mtf1* in mice decreased OA pathogenesis. Authors concluded that the “Zn-ZIP8-MTF1 axis” is required for catabolism that leads to pathogenesis of OA [75]. Whereas the *SLC39A8* gene and flanking regions have no MTF1-binding sites, the *NFKB1* gene does [80]; therefore, the reciprocal regulation between the two adjacent genes *NFKB1* and *SLC39A8* on Chr 4q24—described in detail earlier [44]—likely contributes to the explanation of the “Zn-ZIP8-MTF1 axis” [75].

The Klotho enzyme is encoded by the human *KL* (mouse *Kl*) gene; the gene product is a type-I membrane protein, related to β-glucuronidases; clinically, Klotho appears to improve cognition, kidney disease, and catabolic diseases of aging (reviewed in [81]). Because OA is correlated with increased hypertrophy-associated catabolic matrix-remodeling enzymes and pro-inflammatory cytokines, effects of Klotho were assessed in mouse cartilage homeostasis during both normal cartilage formation and development of OA; *Kl* expression was detected during embryonic limb development, and transiently during chondrogenic differentiation of bone marrow-derived mesenchymal stem cells in culture [82]. Genome-wide transcriptomics of chondrocytes from OA patients revealed that incubation with recombinant-delivered Klotho repressed the expression of nitric-oxide synthase-2 (*NOS2*) and the *SLC39A8*/*MMP13* catabolic-remodeling axis. In chondrocytes, as well as in cartilage of an OA mouse model, chronic IL1B treatment lowered Klotho expression; an intra-articular-secreted *Kl* gene transfer into the intact mouse delayed cartilage degradation in the OA mouse model. These findings suggest a tissue homeostatic function for Klotho in which it protects against onset and progression of OA [82]. These last three paragraphs are summarized in a mechanistic diagram (Fig. 1).

**Fig. 1:** Sequence of steps that describe the first three paragraphs of the section on “*SLC39A8* and the musculoskeletal system,” regarding progression of osteoarthritis. See text for details

Interestingly, matrix metalloproteinases (MMPs) are a family of endopeptidases that are mostly zinc-dependent, but some of them are cobalt-dependent; the metal ion is coordinated to the protein via three ligands. MMPs participate in degradation of various proteins in the ECM. The six classes of MMPs include collagenases, gelatinases, stromelysins, matrilysins, membrane-type MMPs, and other MMPs. These endopeptidases play a role in tissue remodeling during various physiological processes—such as angiogenesis, embryogenesis, morphogenesis, and wound repair—as well as in pathological conditions such as OA, myocardial infarction, fibrotic disorders, and cancer (reviewed in [83]). MMPs are also tightly controlled by posttranslational modifications, including *N*- and *O*-glycosylation (reviewed in [84]). Accordingly, MMPs are involved in virtually every critical life process.

As discussed repeatedly throughout this review, the SLC39A8 transporter is pivotal for the influx of Zn^2+^, Co^2+^, and Mn^2+^ ions into cells of all types. Because Zn (and sometimes Co) are cofactors that are crucial to the function of MMP enzyme activities—and because Mn-dependent posttranslational glycosylation is one means of regulating MMP levels—it therefore becomes obvious that the interplay between SLC39A8 and MMPs is extremely important!

To investigate severe adolescent idiopathic scoliosis, an exome-wide association study was carried out in 457 severe cases vs 987 controls [53]; the *SLC39A8* p.Ala391Thr variant was discovered to be associated with severe adolescent idiopathic scoliosis (*P* = 1.6 × 10^−7^; OR = 2.01). Validation studies in a second cohort (841 cases and 1095 controls) resulted in a combined *P* of 7.0 × 10^−14^ (OR = 1.94). Clinically, the p.Ala391Thr allele was associated with greater spinal curvature, decreased height, increased BMI, and lower plasma Mn levels in the adolescent idiopathic scoliosis cohort. Furthermore, in a mutant *slc39a8* zebrafish line—functional studies revealed decreased Mn influx, vertebral abnormalities, impaired growth, and decreased motor activity [53].

### *SLC39A8* and the eye

Sjögren syndrome is an autoimmune disease that mainly affects exocrine glands; clinically, it is characterized by keratoconjunctivitis sicca and xerostomia [85]. Familial occurrence of Sjögren syndrome appears to be very similar to that seen with systemic lupus erythematosus (SLE) and other autoimmune disorders; the term “primary” Sjögren syndrome is used to indicate when the disorder is present with another autoimmune disease [86], such as SLE. Expression of HLA-DR antigen and intracellular adhesion molecule-1 (ICAM1) in human conjunctival epithelium—is upregulated in patients with dry eyes associated with Sjögren syndrome. SLE-primary-Sjögren syndrome is characterized by autoantibodies, dysregulated B cells, and a notably high female-to-male incidence ratio. By means of a disease-targeted approach to understand if the SLE-primary-Sjögren syndrome displays sex-specific effects, genome-wide genotype and gene expression data in primary B cells from 125 males and 162 females were studied; ten SNVs affecting expression of 16 different genes were found. By analyzing SNV × sex interactions, the *SLC39A8* Ala391Thr variant was identified as one of six SLE-primary-Sjögren syndrome-associated alleles showing differentially expressed regulation in females compared with males [64]. How *SLC39A8* expression might contribute to this gender bias in systemic autoimmune diseases—will require further study. The fact (vide supra) that the *NFKB1* SNV (rs4637409) is an eQTL correlated with downregulation of the neighboring *SLC39A8* gene [44] could be relevant to this study.

### *SLC39A8* and the gastrointestinal tract

Although GWAS have identified more than 200 inflammatory bowel disease (IBD) loci, the genetic architecture of IBD remains poorly understood. In order to identify novel variants associated with IBD, whole-exome sequencing of >10,500 IBD cases and ~ 5720 non-IBD controls revealed an association between Crohn disease (CD) and the *SLC39A8* p.Ala391Thr variant; in two replication cohorts [62], combined meta-analysis was highly significant (*P* = 5.6 × 10^−13^); this finding is consistent with the large GWAS of 42 traits or diseases, mentioned earlier [50]. In addition, in microbiota from 338 mucosal lavage samples from the Mucosal Luminal Interface cohort, association of the p.Ala391Thr variant was examined, using 16S sequencing; it was concluded that the *SLC39A8* risk allele for CD is associated with altered colonic mucosal microbiome composition in both healthy controls (*P* = 0.009) and CD cases (*P* = 0.0009).

Furthermore, microbes depleted in healthy carriers strongly overlapped with those having reduced microbes in CD patients (*P* = 9.2 × 10^−16^) and in overweight individuals (*P* = 6.7 × 10^−16^); these intriguing data suggested that the *SLC39A8* p.Ala391Thr missense variant is somehow associated with a shift in the gut microbiome pattern [62]. However, although a recent study of 291 patients with inflammatory bowel disease and 476 healthy controls did confirm the link between the p.Ala391Thr variant and Crohn’s disease, authors could not replicate association of the risk allele with gut microbiome composition in healthy subjects [87]. Perhaps a much larger cohort might tease out any correlation. The brain-gut-microbiome axis—mentioned earlier [78], but beyond the scope of this review—might apply to other inflammation-based disorders, in which the intestine generates a nidus for problems elsewhere in the body; accordingly, *SLC39A8*, which plays a pivotal role in inflammation [43, 45, 46], is likely linked to disorders such as schizophrenia and OA [vide supra].

### Musings

Throughout this review, in both the earlier mouse studies and the later clinical studies, variability in *SLC39A8* expression was examined—relative to the normal (vs deficient) uptake of Mn^2+^, Zn^2+^, Fe^2+^, or Se^4+^—in terms of beneficial cellular and physiological processes vs deleterious pathophysiology. Many of these mechanistic pathways described are illustrated in Fig. 2.

**Fig. 2:** Molecular mechanisms of ZIP8 transport function and related downstream pathways in various cell organelles. At *far left*, ZIP8 imports Zn^2+^; a cofactor, in the NFκB subunit P65, then inactivates NFκB. Downstream targets SNAIL and CDH1 participate in the immune response, cell morphology, proliferation, and migration. Increased levels of intracellular Zn^2+^ can also activate MTF1 which, in cartilage, enhances catabolic processes—including matrix metallopeptidases (MMP’s) and ADAM metallopeptidases with thrombospondin types (ADAMTS’s) that hydrolyze proteins. At *left center*, Zn^2+^ influx by ZIP8 in the lysosomal membrane elevates cAMP-responsive element-binding protein (CREB), which regulates interferon-γ (INFG) expression involved in the immune response. At *center*, any role for ZIP8-mediated Fe^2+^ uptake has not been studied to date (denoted by the “?”). At *right center*, ZIP8-mediated selenite [(HSeO_3_)^−^] influx likely affects activities of selenoproteins such as glutathione peroxidases-1, -2 (GPX1/2). At *far right*, ZIP8-mediated Mn^2+^ uptake is critical for Mn-dependent enzymes such as mitochondrial manganese-superoxide dismutase (MnSOD) in mitochondria; decreases in both GPX1/2 and MnSOD result in increased oxidative stress. Deficiencies in Mn-dependent enzymes—including β-1,4-galactosyltransferases-1, -2 (B4GALT1/2) in the Golgi body—results in defects in posttranslational glycosylation and almost half of all proteins synthesized in the cell. See text and references cited therein for details

#### Manganese

The divalent cation Mn^2+^ is an essential trace nutrient, as well as cofactor for numerous Mn-containing enzymes belonging to all six major enzyme families, plus several Mn metalloenzymes that carry tightly bound Mn^2+^ cations [88]. Human disorders involving three SLC transporters have been recognized only during this past decade: SLC30A10 deficiency associated with Mn-induced neurotoxicity; and *SLC39A14* and *SLC39A8* mutations correlated with Mn deficiency (reviewed in [89]). To this list can now be added type II (CDG) congenital disorder of glycosylation [17] and Leigh-like mitochondrial disease [20]; both clinical disorders are associated with *SLC39A8* variants of deficient Mn influx, resulting in defective Mn-dependent posttranslational glycosylation of proteins such as transferrin and β-1,4-galactosyltransferase [17, 20, 47]. Because almost half of all proteins are posttranslationally *N*-glycosylated [66]—it should be kept in mind that these *SLC39A8* variants might therefore exert a much farther-reaching impact, contributing to the etiology of many human diseases. There are no known Mn^2+^-containing transcription factors.

#### Zinc

The intracellular nutrient Zn^2+^ is pivotal in homeostasis-related signal transduction pathways, myeloid cell function and host defense against infection [90, 91], cell cycle, cell proliferation, embryonic development, and differentiation [92]. In human and mouse, there are >100 Zn-dependent enzymes [93], >2000 Zn-containing transcription factors [94], and an estimated ~2800 Zn^2+^-binding proteins—corresponding to ~10% of the human proteome [95]. Because these enzymes and transcription factors perform so many critical-life functions throughout development—often employing cell-specific effects on morphogenesis, growth, and differentiation—the embryo’s ability to maintain Zn homeostasis is essential from the single-cell-zygote onward [96]. Defects in Zn uptake that lead to Zn-deficient proteins involved in all types of critical life processes can therefore be life-threatening or fatal, as demonstrated by the mouse and clinical studies described herein.

#### Iron

For Fe^2+^, there are numerous Fe-containing enzymes and other proteins critical to life processes. Dysregulated hematopoiesis during *Slc39a8*(*neo*/*neo*) embryogenesis and fetogenesis [27] is suggestive of an iron-transport defect, although upstream events involving TAL1 and the GATA proteins underscore the pivotal importance of Zn-related transcription factor functions during early hematopoiesis [28]. Whereas there are a few Fe-containing transcription factors in prokaryotes [97], no Fe-containing transcription factors have been identified in eukaryotes.

#### Selenium

The micronutrient Se^4+^ is essential in human and mouse for ~25 Se-containing proteins, the majority of which exhibit anti-oxidative activities; selenoproteins are involved in numerous physiological functions—e.g., redox regulation and signaling, thyroid hormone metabolism, selenocysteine synthesis, Se transportation and storage, protein-folding, as well as preventing or slowing down inflammation, cancer and aging [98]. Se must be intracellular in order to carry out these functions, and it is indeed intriguing that the ZIP8- and Zn-dependent uptake of selenite (HSeO_3_^−^) appears to be among the principal mechanisms by which Se enters the cell [15]. Clinical Se deficiency can lead to cardiovascular and myodegenerative diseases, infertility, premature births, and osteochondropathy (Kashin-Beck disease). Recent transcriptional analyses of Kashin-Beck disease patients have identified novel cellular pathways that might be related to transcriptional regulation by Se [99], although currently there are no known Se-containing transcription factors.

#### Cobalt

For Co^2+^, human embryonic kidney HEK293T cell cultures transfected with *SLC39A8* cDNA resulted in greater uptake of not only Mn^2+^, Zn^2+^, and Fe^2+^—but also Co^2+^ [13]; although, to date, nothing substantial has been reported vis-a-vis ZIP8-mediated Co uptake, this essential nutrient is normally taken up in the diet and worthy of mention. The organic form of Co is a necessary component of vitamin B_12_, which participates in amino acid synthesis, nerve cell proteins, and neurotransmitters; either vitamin B_12_ excess or deficiency can lead to human disorders [100]. Under physiological conditions, vitamin B_12_ bound to the gastric intrinsic factor is internalized in the ileum by a highly specific receptor complex, comprising cubilin (CUBN) and amnion-associated transmembrane protein (AMN); after leaving the ileum, general cellular uptake of the vitamin B_12_ complex from the blood is mediated by transcobalamin-2 (TCN2), whereas kidney tubular reabsorption of vitamin B_12_ requires LDL receptor-related protein-2, LRP2 [101]. Any critical role of ZIP8-mediated uptake of Co will require further study; for example, in *SLC39A8*-deficient patients suffering from schizophrenia or Parkinson disease, would Co^2+^-mediated (vitamin B_12_-mediated) nerve cell protein and neurotransmitter defects contribute to these neurological disorders? There are no known Co-containing transcriptional factors.

#### Cell-type specificity of SLC39A8-mediated functions

Do ZIP8-mediated functions primarily reflect Mn, Zn, Fe, Se, or Co uptake—or do they depend on specificity of the organ, tissue, or cell-type? Curiously, six human *SLC39A8* variants have been putatively correlated with many developmental disorders, hypomanganesemia, hypermanganesuria, and glycosylation deficiency [17, 20, 47], whereas just one variant (p.Ala391Thr) is associated with striking pleiotropy of at least 22 other traits (Table 1). An understanding of these observations will require further study—perhaps including three-dimensional modeling, structural biology, and studies of physical (Mn, Zn, Fe, Se, and Co) ion-binding properties of each ZIP8 transporter variant. One promising approach would be to expand on the elegant definitive studies [19, 68], in which constructed mutant alleles were transfected into human cell cultures, comparing Mn uptake by each mutant with consensus *SLC39A8* cDNA. We would propose, however, that cDNA constructs encoding each of the seven protein alterations (Table 1) be *individually* introduced into numerous cell types: e.g., plutipotent ES cells, monocytes or other cells of myeloid origin, cardiomyocytes, hepatocytes, renal tubular epithelium, lung epithelial cells, megakaryocytes, CNS neurons, chondrocytes, conjunctival epithelial cells, and gastrointestinal epithelial cells (Fig. 3). In each cell type, each *SLC39A8* variant should be tested separately against consensus *SLC39A8* cDNA for Mn, Zn, Fe, Se, and Co uptake. Would any substantial differences in metal ion uptake be discovered, depending on the cell type?

**Fig. 3:** Summary of all organs and systems in which *SLC39A8* variants have been associated with clinical disorders (to date)—discovered principally by GWAS and whole-exome sequencing studies. The “?” denotes additional organs or system in studies that have not yet been published

## Conclusions

Expression of the *Slc39a8*-encoded ZIP8 transporter of cation uptake is detectable in mouse gastrula and visceral endoderm at GD7.5 during embryogenesis; *Slc39a8* expression has been suggested to be used as an indicator of cell differentiation in pluripotent ES cells. Therefore, it comes as no surprise that human *SLC39A8* variants reveal extreme pleiotropy—with reports of associations with clinical disorders in numerous organ, tissue and cell types, physiological processes, and quantitative traits (Fig. 3 and Table 1): *congenital birth defects* (mental retardation, developmental delay, cerebellar and cerebral atrophy, cranial asymmetry, severe seizures, severe infantile spasms with hypsarrhythmia, disproportionate dwarfism, deformed skull, profound psychomotor retardation and developmental delay, hypotonia and dystonia, hearing loss, strabismus, short limbs, short stature, failure to thrive); *the immune system* (innate immune response, protection against inflammation, increased risk of allergy); *the cardiovascular system* (lower serum HDL-Chol levels, increased risk of coronary artery disease, hypotension, smoking-induced atherosclerotic plaques, acute coronary syndrome, cardiovascular death); *liver* (Mn-deficient hypoglycosylation, Leigh-like mitochondrial disease, increased BMI, inflammation and fibrosis]; *kidney* (hypotension, elevated NT-proBNP levels); *lung* (innate immune response, anti-inflammatory); *the coagulation system* (increased VWF plasma levels); *central nervous system* (elevated risk of schizophrenia, Parkinson disease, cerebrovascular disease); *musculoskeletal system* (participation in osteoarthritis, increased risk of severe adolescent idiopathic scoliosis, decreased height); *the eye* (myopia, SLE-primary-Sjögren syndrome); and *gastrointestinal tract* (inflammatory bowel disease, Crohn disease).

In virtually all cases, deficiencies in *SLC39A8* expression (decreased metal ion uptake) are detrimental, i.e., SLC39A8-mediated cation influx is beneficial to all cells. Normal SLC39A8 function is good; SLC39A8 deficiency results in various undesirable diseases or quantitative traits. The one apparent “exception” is that deficient *SLC39A8* expression is associated with downregulation of matrix-degrading enzyme activities—resulting in failure to inhibit chondrocyte degeneration and OA [65, 75]. However, the most likely explanation is that cytokine-induced chronic inflammation, by way of KLOTHO suppression (Fig. 1), is the primary unfavorable signal that initiates OA; the inflammatory process then also stimulates *SLC39A8* expression to combat the disease by increasing Zn influx. Hence, ZIP8 is not *the cause* of this pathology, but is merely swept up as an “innocent bystander,” doing its best to combat all forms of inflammation, which—in this case—includes chronic OA.

Finally, it should be mentioned that the *SLC39A8* gene should be regarded as “an unlikely drug target,” if one wishes to treat any of the disorders described herein. Because *SLC39A8* is expressed in pluripotent ES cells and developmentally in every cell type onward into adulthood, this means ZIP8-mediated cation influx is expressed, or capable of being expressed, in virtually every cell type in the body. To target this gene (or mRNA or protein) with any new drug, and call *SLC39A8* a “druggable target”—would require highly specific targeting to one cell type, while being assured that all other cell type ZIP8 “off-targets” are not inadvertently blocked or stimulated.

This is one difference between *SLC39A8* and, say, *SLC39A4*—mutations in which are well-known to cause acrodermatitis enteropathica, zinc-deficiency (AEZ) type [102]. Whereas *SLC39A8* contributes as one of many dozens or hundreds of genes, discovered by GWAS, that are associated with various complex diseases and quantitative traits—*SLC39A4* is not expressed in pluripotent ES cells and, consequently, mutations that cause ZIP4 deficiency result in such diseases as AEZ, inherited as a recessive Mendelian trait (i.e., caused by only one or just a few genes). Therefore, targeting *SLC39A8* to treat schizophrenia or coronary is highly problematic, whereas treatment of AEZ (e.g., Zn supplementation) can be relatively straightforward.

What will the future hold? It will be exciting to learn about discoveries of additional clinical disorders correlated with *SLC39A8* variant alleles and their associated deficiencies in uptake of intracellular Mn^2+^, Zn^2+^, Fe^2+^, Se^4+^, and probably also Co^2+^.

In a very recent study on the genetic architecture of alcoholism — a meta-analysis of more than 480,800 people of European descent identified 46 novel common genetic loci and investigated their potential functional importance, using magnetic resonance imaging and gene expression studies [103]; one of the genes highest on the list of statistical significance was the SLC39A8 p.Ala391Thr variant (P = 1.3 × 10–15). Authors noted that many of their identified genetic pathways are not only associated with alcohol consumption, but also shared with neuropsychiatric disorders such as schizophrenia.

## Data Availability

Data-sharing not applicable to this review.

## Abbreviations

AAV: Adeno-associated virus
ABCs: Members of the ATP-binding cassette transporter group
*Ace2*: Angiotensin-1-converting enzyme-2 (mouse) gene
ADAMTS: “A disintegrin and metalloproteinase with thrombospondin motifs” group of enzymes
AEZ: Acrodermatitis enteropathica caused by zinc-deficiency
*Alb>Cre>Slc39a8*(*fl*/*fl*): Hepatocyte-specific *Slc39a8* conditional knockout mouse line
AMN: Amnion-associated transmembrane protein
ANP: Atrial natriuretic peptide
*Apoe*: Apolipoprotein-E (mouse) gene
B6: C57BL/6J inbred mouse
BCL2: BCL2 apoptosis regulator
BMI: Body mass index
*BTZIP8–3*: BAC-transgenic mouse line carrying five *Slc39a8* genes
C/EBPβ: CCAAT/enhancer-binding protein-beta
CASPASE 3: Caspase-3 apoptosis-related cysteine protease
Cd: Cd^2+^ cadmium ion
CD: Crohn disease
TCN2: Transcobalamin-2
CDG: Congenital disorder of glycosylation
CDH1: Cadherin-1 (E-cadherin)
CDK: Chronic kidney disease
cM: CentiMorgans
CNS: Central nervous system
Co: Co^2+^ ion
COL1A2: Collagen type-I α2 chain
COMPASS: Complex of proteins associated with a trithorax-related SET domain protein
*COX18*: Cytochrome c oxidase assembly factor-18
cT1-MRI: corrected T1-magnetic resonance imaging
CUBN: Cubilin
D2: DBA/2 J inbred mouse
DCM: Dilated cardiomyopathy
*DNAH*: Dynein heavy chain-5 axonemal gene
ECM: Extracellular matrix
eQTL: Expression quantitative trait locus
ES cells: Embryonic stem cells
Fe: Fe^2+^ ferrous ion
FVIII: Coagulation factor-8
GD: Gestational day
GWAS: Genome-wide association study (or studies)
HCO_3_^−^: Bicarbonate ion
HDL: High-density lipoprotein
HLA-DR: Major histocompatibility complex, class II, DR group
HSeO_3_^−^: Selenite, containing Se^4+^ ion
IBD: Inflammatory bowel disease
ICA: Independent component analysis
ICAM1: Intracellular adhesion molecule-1 (also known as cluster of differentiation-54; CD54)
IFNG: Interferon-γ
*IKBKB*: Inhibitor of nuclear factor kappa B kinase subunit beta
*IKBKE*: Inhibitor of nuclear factor kappa B kinase subunit beta
IL10 & IL8 & IL6 & IL1B: Interleukin proteins
IκB or IKK: Inhibitor of nuclear factor kappa B kinase [a complex of four genes including CHUK (component of inhibitor of nuclear factor kappa B kinase complex)]
*KL*: Klotho gene
LDL- and HDL-Chol: LDL- and HDL-cholesterol
LDL: Low-density lipoprotein
LPS: Lipopolysaccharide
LRP2: LDL-receptor-related protein-2
LVNC: Left ventricular noncompaction
MAF: Minor allele frequency
MAPK1: Mitogen-activated protein kinase-1
Mb: Megabases
MEFs: Mouse embryonic fibroblasts
miRNA: Micro-RNA
MMP3 & MMP9 & MMP12 & MMP13: Matrix metallopeptidases
Mn: Mn^2+^ manganous ion
MnSOD: Manganese-superoxide dismutase-2 encoded by *SOD2* gene
MTF1: Metal regulatory transcription factor-1
NAFLD: Non-alcoholic fatty liver disease
NASH: Non-alcoholic steatohepatitis
NFκB complex: Nuclear factor kappa-light-chain-enhancer of activated B cells which includes *NFKB1*-encoded protein NFKB1
*NOS2*: Nitric-oxide synthase-2 gene
*Npr3*: Natriuretic peptide receptor-3 (mouse) gene
NT-proBNP: NH_2_-terminal pro-B-type natriuretic peptide
OA: Osteoarthritis
PHA: Phytohemagglutinin
*PLCB1*: Phospholipase-C-beta-1 gene
RI: Recombinant inbred
rvZIP8: Stably transfected MEFs containing ZIP8 cDNA via retroviral infection
*Sglt2 > Cre > Slc39a8*(*flox*/*neo*): Renal tubular epithelium-specific *Slc39a8* conditional knockout mouse
siRNA: Small interfering RNA
SLC: Solute-carrier transporters
SLC39A8: Encoded protein of human *SLC39A8* and mouse *Slc39a8* gene
*SLC39A8*: Human gene encoding the metal ion influx transporter ZIP8—(also when referring to the generic gene in all vertebrates)
*Slc39a8*: Mouse gene encoding ZIP8
*Slc39a8*(*neo*/*neo*): Knockdown mouse line expressing ~15% of wild-type *Slc39a8* mRNA and ZIP8 protein in all tissues examined
SLE: Systemic lupus erythematosus
SNAIL2: Snail transcriptional repressor-2
SNVs: Single-nucleotide variants
TAL1: T cell acute lymphocytic leukemia protein-1
TBK1: TANK-binding kinase-1)
TGFβ3: Transforming growth factor beta-3 encoded by *TGFB3* gene
TNF: Tumor-necrosis factor
*UBC>Cre>ERT2>Slc39a8*(*fl*/*fl*): Inducible global-knockout of *Slc39a8* mouse line
UPF3A: UPF3A regulator of nonsense-mediated mRNA decay
VWF: Von Willebrand factor
ZIP8: Trivial or jargon name for the transporter “zinc- and iron-related protein-8”
Zn: Zn^2+^ zinc ion
